The article "HMGB1 mediates lipopolysaccharide-induced inflammation via interacting with GPX4 in colon cancer cells" was published in 2020. Journal: Cancer Cell Int.

# HMGB1 mediates lipopolysaccharide-induced inflammation via interacting with GPX4 in colon cancer cells

**DOI:** 10.1186/s12935-020-01289-6

**Published:** 2020-05-29

**Authors:** Yuhan Yang, Ling Yang, Sheng Jiang, Ting Yang, Jingbin Lan, Yun Lei, Hao Tan, Kejian Pan

**Affiliations:** 1 School of Bioscience and Technology, Chengdu Medical College, Chengdu, 610500 Sichuan People’s Republic of China; 2 School of Basic Medical Sciences, Chengdu Medical College, Chengdu, People’s Republic of China; 3 Ministry of science and technology, Second Affiliated Hospital of Chengdu Medical College (China National Nuclear Corporation 416 Hospital), Chengdu, People’s Republic of China; 4 Department of pathology, Yiyang Central Hospital, Yiyang, 413000 Hunan People’s Republic of China

**Keywords:** HMGB1, GPX4, p-p65, ROS, Inflammation, Colon cancer

## Abstract

**Background:**

Inflammation is one of a main reason for colon cancer progression and poor prognosis. The high-mobility group box-1 (HMGB1) and glutathione peroxidase 4 (GPX4) are responsible for inflammation, but the relationship between HMGB1 and GPX4 remains unknown about inflammation in colon cancer.

**Methods:**

RT-qPCR was carried out to investigate the expression of IL1β, IL6 and TNFα in colon cancer cells stimulated with LPS or siHMGB1. To observe the relationship between HMGB1, GPX4 and inflammation or ROS, Western blot assays were adopted. Pull-down, CoIP and immunohistochemistry assays were performed to further investigate the molecular mechanisms of HMGB1 and GPX4 in colon cancer.

**Results:**

We report that HMGB1 mediates lipopolysaccharide (LPS)-induced inflammation in colon cancer cells. Mechanistically, acetylated HMGB1 interacts with GPX4, negatively regulating GPX4 activity. Furthermore, by utilizing siHMGB1 and its inhibitor, our discoveries demonstrate that HMGB1 knockdown can inhibit inflammation and reactive oxygen species (ROS) accumulation via NF-kB.

**Conclusion:**

Collectively, our findings first demonstrate that acetylated HMGB1 can interact with GPX4, leading to inflammation, and providing therapeutic strategies targeting HMGB1 and GPX4 for colon cancer.

## Background

Colon cancer is the malignant carcinoma and the third most common cancer worldwide leading to causes of deaths [1]. The early stage of colon carcinoma can be treated by using surgical extraction, radiotherapy and drugs. Colon cancer or infectious agents can be as a danger molecule in our tissue, and then immune system cells respond to the damage and intent to eliminate the danger [2, 3]. These immune cells produce pro-inflammatory cytokines IL1β, IL6 and TNFα to increase strength of the response against danger [4]. Previous study has shown that the anti-inflammatory drugs are associated with the reduced incidence and the metastasis rat in the colon cancer [5]. Inflammation is one of the main reasons and critical incidents for cancer progression and poor prognosis, particular in colon cancer [6]. Thus the molecular mechanisms between colon cancer and inflammation demand for further study in detail which can provide the treatment strategies for colon cancer.

HMGB family, including HMGB1, HMGB2 and HMGB3, have been studied for the past decade as the nuclear components important for transcription and chromatin structure [7]. HMGB1, also termed HMG1 and amphoterin, is most abundant member of HMGB family of the DNA-binding proteins [8–10]. Normally, HMGB1 protein exist in cell nucleus; when it is released to the extracellular space upon the cell damage, it becomes an immune-inflammatory factor [11–13]. In general, the stimulation of cells by cytokines, lipopolysaccharide (LPS) or hypoxia enables HMGB1 export from nucleus to cytoplasm or the extracellular space, and acetylation of HMGB1 has been suggested to regulate its intracellular shutting in cells [14, 15]. Evidences have shown that the extracellular HMGB1 can be as a mediator of inflammation and tissue regeneration [8, 16]. HMGB1 is closely related to many inflammatory diseases, such as ischemia of liver and kidney, hepatitis, arthritis, stroke, ischemia of liver and kidney, sepsis, and systemic lupus erythematosus [17–19]. Yet, the link between HMGB1 and inflammation in colon cancer remains unclear, and then we have proposed the hypothesis that HMGB1 mediated the inflammation in colon cancer.

GPX (glutathione peroxidase) is the intracellular anti-oxidant enzyme responsible for reducing peroxides. GPX4, a member of the GPxs family, also called phospholipid hydroperoxide glutathione peroxidase (PHGPx), is considered one of the important antioxidant enzymes in the mammals [20–22]. GPX4 is especial among the GPX family in that it has a unique affinity for membrane-bound substrates such as the phospholipids and cholesterol hydroperoxides [23–25], directly reducing the membrane-bound phospholipid hydroperoxides in the situ and protecting against damage. Lipid hydroperoxides are implicated in variety of pathophysiological processes, including inflammation. Besides being able to repair lipid peroxides as the antioxidant enzyme, GPX4 can also regulate cytokine signaling [26]. GPX4 is identified as a central regulator of the ferroptosis, a newly discovered the iron-dependent cell death and latest addition to list of the surprises [27, 28]. However, just like HMGB1 as a mediator of inflammation, GPX4 can be also responsible for inflammation, the connections of HMGB1 and GPX4 are not currently known.

Here we report that HMGB1 mediates LPS-induced inflammation in colon cancer cells. LPS was used to mimic the danger and then stimulate SW480 and HCT116 colon cells. In order to explore the inflammation under LPS stimulated conditions, we detected the mRNA levels of pro-inflammatory cytokines IL1β, IL6 and TNFα. Our results revealed that HMGB1 can bind with GPX4, thus mediating the occurrence and development of inflammation induced by LPS. Our discoveries provide a novel molecular mechanism of inflammation in colon cancer cells and the therapeutic strategies for colon cancer.

## Materials and methods

### Plasmid construction and siRNA

cDNA encoding GPX4 was synthesized and cloned into the pcDNA3.1(+) expression vector (Invitrogen) using the segment and fusion PCR. Meanwhile, To silence the expression of HMGB1 in SW480 and HCT116 cells, siHMGB1 was purchased from Santa Cruze. After seeding into the 6-well plates, the siHMGB1 or pcDNA3.1-GPX4 were transfected into SW480 and HCT116 cells utilizing Lipofectamine 2000 transfection reagent (Invitrogen, Carlsbad, CA, USA). The protein levels of HMGB1 and GPX4 were detected after transfection for 48 h by western blot.

### Cell culture and treatment

SW480 and HCT116 colon cancer cells were maintained in School of Biological Science and Technology, Chengdu Medical College. The cells were cultured in the Dulbecco’s modified Eagle medium (DMEM) containing 10% fetal bovin serum (FBS) and then transfected with the jetPRIME (#114-15, SA, France), thus incubated in the 5% CO_2_ incubator at 37 °C. For treatment, after transfetion, the cells were pretreated utilizing various does of GL (glycyrrhizin) (Sigma, St. Louis, MO, USA) (1 mmol/L) for 12 h and stimulated with 1 μg/ml LPS for 6 h. Then cells were harvested and analyzed using the appropriate antibodies. All experiments were repeated for three times.

### Quantitative real-time PCR (qRT-PCR) assay

For quantitative real-time PCR, the cells under various treatment were collected by using TRIzol (Invitrogen) to extract the total RNA. And then The cDNA was synthesized by utilizing the SuperScript II First Strand Synthesis System (Invitrogen). The qRT-PCR was performed to quantify the IL-1β, IL-6 and TNF-α transcript levels by using the specific primers. The β-actin, housekeeping gene, was an internal standard to calculate the target gene relative expression using the 2 − ΔΔCT formula. qRT-PCR was performed by the quantitative real-time PCR system (BioRad, Hercules, CA, USA), with the first denaturation step, followed with the 40 cycles containing denaturaion, annealing and extension.

### Immunoprecipitation (IP) and western blot

For IP assay, the cells were lysed by using the protein extraction buffers (PP1801, Bioteke, China) containing the protease inhibitor (04693116001, Roche, Switzerland) after transfected with siHMGB1 and pcDNA3.1-GPX4 for 48 h. The extracted protein was immunoprecipitated with the specific antibody and protein A + G agarose beads (P2012, Beyotime, China). For western blot, equal amounts of proteins were separated with SDS-PAGE and subsequently transferred to the PVDF membrane, then detected using primary antibody and the horseradish peroxidase-conjugated secondary antibodies. After that, the special immunoreactive bands were detected with chemiluminescence western blot detection system (WBKLS0100, Millipore, USA).

### ROS detection by fluorescence microscope

To detect the intracellular ROS levels in SW480 and HCT116 cells, Reactive Oxygen Species Assay Kit (S0033, Beyotime, China) was used. The cells were seeded in a 24-well culture plate at a density of 2 × 10^5^ cells/well. The reagents freely enter into the cells and then become highly fluorescent after being oxidized by the ROS. LPS, siHMGB1 and pcDNA3.1-gpx4 administration, the medium of culture plate was discarded, and then cells were washed using PBS (phosphate-buffered saline). Subsequently, the colon cells were incubated with 10 μM reagents for 20 min at 37 °C, and the results were analyzed by fluorescence microscope.

### GPX4 activity assay

GPX4 activity assay was performed using the Glutathione Peroxidase Activity Colorimetric Assay Kit (Bioversion, catalog: #K762-100) according to manufacturer’s instructions. Colon cancer cells on ice in 0.2 ml cold assay buffer; Centrifuge at 10,000*g* for 15 min at 4 °C; Collect the supernatant for assay and store on ice. Serum can be tested directly. We suggest testing several doses of your sample to make sure the readings are within the standard curve range. The cellular extracts of colon cancer cells treated with the DMSO or the indicated concentrations of LPS for 6 h were then prepared according to manufacturer’s instructions. GPX activity assay was assessed via measuring changes in absorbance at 340 nm to the NADPH standard curve.

### Immunohistochemistry

Colon cancer tissues were sliced at the thickness of 4 μm, and then sections were placed on the silane-coated slides and deparaffifinized. Antigen retrieval based on heat, the endogenous peroxidase block with 3% hydrogen peroxide, and then blocking were performed using normal sera. The used primary antibodies were HMGB1, GPX4, and p-p65. Specimens with the antibodies were incubated for overnight at 4 °C. The visual color was performed by using the diaminobenzidine (DAB; Nichirei Bioscience, Japan).

### Statistical analysis

The whole data were repeated at least three separate times, and were expressed as the mean ± SD with the GraphPad Prism 7.0 software. The statistical analyses were analyzed using the SPSS version 17.0. For the comparison, differences were determined with the Student’s test among the experimental groups. Statistical significance was considered as the Values of P < 0.05.

## Results

### LPS increases inflammation in HMGB1-dependent manner

To explore the role of LPS in inflammation, we firstly investigate mRNA levels of pro-inflammatory cytokines IL1β, IL6 and TNFα by using qRT-PCR assay. As shown in Fig. 1a, LPS elevated the mRNA levels of IL1β, IL6 and TNFα after LPS treatment for 48 h in SW480 and HCT116 cells. Evidences have shown that HMGB1 is a therapeutic target and NF-kB plays a crucial role in inflammatory response [8, 27], so we next confirmed whether HMGB1 contributed to inflammation induced by LPS in SW480 and HCT116 cells. The western blot results indicated LPS increased the HMGB1, p-IKBα and p-p65 protein expression, when siHMGB1 were introduced, this effect was weakened (Fig. 1b). Then we performed real-time PCR and the results showed HMGB1 knockdown effectively decreased the IL1β, IL6 and TNFα mRNA levels increased by LPS (Fig. 1c). And the change of HMGB1 levels may be in extracellular space, then we detected the extracellular HMGB1 and the results showed no significant concentration of HMGB1 were observed in extracellular space after LPS treatment for 0 h to 72 h (Fig. 1d). Suggesting that LPS increases inflammation in HMGB1-dependent manner.

**Fig. 1:** LPS increases inflammation in HMGB1-dependent manner. **a** Quantitative real-time PCR results showed that LPS elevated the mRNA levels of pro-inflammatory cytokines IL1β, IL6 and TNFα after LPS treatment for 48 h in SW480 and HCT116 cells. **b** Western blot results indicated LPS increased the HMGB1, p-IKBα and p-p65 proteins expression in SW480 and HCT116 cells, when siHMGB1 were introduced, this effect was weakened. **c** qRT-PCR results revealed that siHMGB1 effectively decreased the IL1β, IL6 and TNFα mRNA levels increased by LPS. **d** Extracellular HMGB1 were detected and the results showed no significant change of HMGB1 were observed in extracellular space after LPS treatment for 0 h to 72 h

### HMGB1 regulates inflammation via ROS-mediated

As we know that reactive oxygen species (ROS) and inflammation are tightly linked [30, 31], we want to know whether ROS was involved in inflammation in SW480 and HCT116 cells. The results demonstrated that LPS could promote ROS accumulation (Fig. 2a). Then we treated cells with ROS scavenger NAC (N–acetyl–cysteine) and harvested for western blot, the results revealed NAC suppressed the p-IKBα and p-p65 protein levels increased by LPS (Fig. 2b). Interesting, in cells treated with siHMGB1 to investigated the links between HMGB1 and ROS, siHMGB1 significantly suppressed the ROS accumulation (Fig. 2c). Next we detected the levels of GSH (Glutathione), a antioxidant, and the results showed that LPS effectively repressed the GSH levels. In contrast, siHMGB1 could increase the GSH levels (Fig. 2d). Taken together, above results suggested that HMGB1 regulates inflammation via ROS-mediated.

**Fig. 2:** HMGB1 regulates inflammation via ROS-mediated. **a** To investigate whether ROS was involved in inflammation, we detected the ROS levels in SW480 and HCT116 cells and the results demonstrated that LPS could promote ROS accumulation. **b** The cells treated with ROS scavenger NAC and harvested for western blot, the results showed that NAC inhibited the protein levels of p-IKBα and p-p65 stimulated by LPS. **c** In cells treated with siHMGB1 to investigated ROS levels, siHMGB1 significantly suppressed the ROS accumulation. **d** The levels of GSH were detected and the results showed that LPS effectively repressed the GSH levels. In contrast, siHMGB1 increased the GSH levels. ROS, reactive oxygen species; NAC, N–acetyl–cysteine; GSH, Glutathione

### HMGB1 interacts with GPX4

GPX4 is one of the most important antioxidant enzymes, directly reducing the membrane-bound phospholipid hydroperoxides and protecting against damage [20]. Previous studies have shown HMGB1 and GPX4 are associated with inflammation, then we identify the relationship of HMGB1 and GPX4. Firstly, the cells were transfected with siHMGB1 to observe the changes of GPX4 activity, and the results showed siHMGB1 could increase the GPX4 activity which was repressed by LPS (Fig. 3a). The further IP results indicated that HMGB1 could interact with GPX4 in a dose-dependant manner in SW480 and HCT116 cells with LPS stimulated, but cells without LPS treatment failed to observe the interaction between HMGB1 and GPX4 (Fig. 3b). We constructed over-expression vectors of GPX4, which were injected into SW480 and HCT116 cells. The western blot results showed that the GPX4 protein expressions were up-regulated in pcDNA3.1-GPX4 groups (Fig. 3c). To confirm the function of GPX4, we detected the ROS and MDA (malondialdehyde) levels. And the results indicated GPX4 could suppress the ROS accumulation and MDA levels, which were increased by LPS (Fig. 3d, e).

**Fig. 3:** HMGB1 interacts with GPX4. **a** The cells were transfected with siHMGB1 to observe the changes of GPX4 activity, and the results showed that siHMGB1 could increase the GPX4 activity which was repressed by LPS. **b** IP results indicated that HMGB1 interacted with GPX4 in a dose-dependant manner with LPS simulated, but cells without LPS treatment failed to observe this interaction. **c** Over-expression vectors of GPX4 were constructed to be injected into SW480 and HCT116 cells. Western blot results showed that GPX4 protein expressions were up-regulated in pcDNA3.1-GPX4 groups. To investigate the function of GPX4, we detected the ROS and MDA levels and the results indicated that GPX4 could suppress the ROS accumulation (**d**) and MDA levels (**e**), which were elevated by LPS. MDA, malondialdehyde

### Effects of LPS on HMGB1 translocation

Studies have revealed LPS stimulates cells and can enable HMGB1 release towards cytoplasm, then we examined this effect in SW480 and HCT116 cells. Western blot results indicated that LPS increased HMGB1 expression in cytoplasm but decreased the nuclear HMGB1 protein levels (Fig. 4a). While when inhibitor (Gly, Glycyrrhizic acid) of HMGB1 was introduced, HMGB1 translocation was blocked (Fig. 4b), and IP results revealed Gly attenuated the interaction between HMGB1 and GPX4 (Fig. 4c). Next we investigated whether Gly have an impact on ROS levels and NF-kB. As shown in Fig. 4d, e, Gly significantly suppressed the ROS levels and p-IKBα and p-p65 protein levels increased by LPS, suggesting that LPS promoted HMGB1 migrated from the nucleolus to the cytoplasm to affect the ROS accumulation and mediated inflammation.

**Fig. 4:** Effects of LPS on HMGB1 translocation. **a** Western blot were performed to observe HMGB1 translocation and the results showed that LPS increased HMGB1 expression in cytoplasm but decreased the nuclear HMGB1 protein levels in SW480 and HCT116 cells. **b** When inhibitor Gly of HMGB1 was introduced, western blot results demonstrated that HMGB1 translocation was blocked. **c** IP results revealed that Gly attenuated the interaction between HMGB1 and GPX4. We investigated whether Gly have an impact on ROS levelsand NF-kB and the results showed that Gly significantly suppressed the ROS levels (**d**) and p-IKBα and p-p65 protein levels (**e**) increased by LPS. Gly, Glycyrrhizic acid

### Acetylated HMGB1 contributes to interact with GPX4 to regulate ROS levels and inflammation

We have provided the data that HMGB1 interacted with GPX4 with LPS treatment, we next would like to know whether acetylated HMGB1 interacted with the GPX4. Pulldown assay was performed to further prove this interaction that HMGB1 could interact with the GPX4 in SW480 and HCT116 cells (Fig. 5a). Then IP results revealed LPS elevated the acetylation level of HMGB1, acetylated HMGB1 was responsible for this interaction (Fig. 5b).

**Fig. 5:** Acetylated HMGB1 contributes to interact with GPX4 to regulate ROS levels and inflammation. **a** Pulldown assay was performed to further prove that HMGB1 interacted with the GPX4 in SW480 and HCT116 cells. **b** IP results revealed that LPS elevated the acetylation levels of HMGB1 and acetylated HMGB1 was responsible for the interaction between HMGB1 and GPX4. **c** Western blot results indicated leptomycin B (an inhibitor of nuclear export) prevented HMGB1 translocation. **d** Western blot results showed that Res administration blocked HMGB1 nucleocytoplasmic translocation with increased Sirt1 expression. **e** IP results showed Res weakened the interaction of HMGB1 and GPX4. Our data sought to examined the connection between Res and ROS levels/NF-kB and the results indicated that Res effectively inhibited the levels of ROS (**f**) and p-IKBα and p-p65 protein expressions (**g**) elevated by LPS. Res, resveratrol

Next we used leptomycin B, an inhibitor of nuclear export, to prevent HMGB1 nuclear export for western blot, and the results indicated that leptomycin B administration blocked HMGB1 translocation (Fig. 5c). Evidences have showed that resveratrol (Res) treatment inhibited the translocation of HMGB1 into the cytoplasm and Sirt1 contribute to HMGB1 nucleocytoplasmic translocation pathway [32, 33]. Western blot showed that Res treatment prevented HMGB1 translocation with increased Sirt1 expression (Fig. 5d). Meanwhile, IP results showed Res weakened the interaction of HMGB1 and GPX4 (Fig. 5e). Then our data sought to examined the connection between Res and ROS levels/NF-kB, and the results indicated that Res effectively inhibited the levels of ROS and p-IKBα and p-p65 protein expressions elevated by LPS (Fig. 5f, g). Our results showed that LPS increased acetylated HMGB1 levels to interact with GPX4 and Res blocked HMGB1 nucleocytoplasmic translocation.

### HMGB1 and GPX4/p-p65 correlation analysis in colon cancer tissues

Above results have proved the connection between HMGB1, GPX4 and p-p65 in SW480 and HCT116 cancer cells, we thereby explored the HMGB1, GPX4 and p-p65 correlation in colon cancer tissues. We performed immunohistochemistry and analyzed the expression and correlation of HMGB1, GPX4 and p-p65 by tissue microarray containing 50 pairs of colon tumor tissues, the clinicopathological data of the patients in the study were in Table 1. And we found that HMGB1, GPX4 and p-p65 were expressed in the tumor tissues (Fig. 6a). And then correlation analysis showed that HMGB1 was positively correlated with GPX4 and p-p65 (Fig. 6b), providing the therapeutic target for colon cancer. Subsequently, by using of cancer and adjacent tissue from seven patients with colon cancer, we found that acetylated HMGB1 and p-P65 expression were increased, the results further demonstrated acetylated HMGB1 and p-P65 expression mediate inflammation in colon cancer (Fig. 6c).

**Table 1:** Clinicopathological data of the patients in the study

Characteristic	Patients (n)
Gender	
Male	17 (56.7%)
Female	13 (43.3%)
Age	
Mean	56
≤ 56	14 (46.7%)
> 56	16 (53.3%)
UICC stage	
I	6 (20%)
II	15 (50%)
III	9 (30%)
TMN N stage	
N0	28 (93.3%)
N1	2 (6.7%)
N	0

**Fig. 6:** HMGB1 and GPX4/p-p65 correlation analysis in colon cancer tissues. We performed immunohistochemistry and analyzed the expression and correlation of HMGB1, GPX4 and p-p65 by tissue microarray containing 50 pairs of colon tumor tissues, and found that HMGB1, GPX4 and p-p65 were expressed in the tumor tissues (**a**) and correlation analysis showed that HMGB1 was positively correlated with GPX4 and p-p65 (**b**). **c** Western blot indicated acetylated HMGB1 and p-P65 expression were increased by using of cancer and adjacent tissue from seven patients with colon cancer. Scale bars: 50 μm

## Discussion

Colon cancer is malignant tumor leading causes of deaths and a challenge to the clinicians throughout the world [1]. Evidences have shown that inflammation is a critical reason for colon cancer progression and poor prognosis [6]. Thus the clarification of this mechanisms for colon cancer treatment is extremely urgent. In this study, our immunoprecipitation results showed that HMGB1 can interact with GPX4 in both colon cancer cells, thus leading to ROS accumulation and inflammation stimulated by LPS, identifying the novel mechanism for colon cancer therapy.

Studies have shown that LPS can induce inflammation and oxidative stress [34–36]. To verify LPS-stimulated cell models, we investigated the effects of LPS on the mRNA level of pro-inflammatory cytokines *IL1β*, *IL6* and *TNFα* and ROS levels in SW480 and HCT116 cells, and then our data determine this effect. As a inflammation mediator and a biomarker and drug target, HMGB1 is currently related to many inflammatory diseases [37]. In this study, the results showed that siHMGB1 suppress inflammatory gens mRNA and ROS levels, in contrast, elevated the GSH level, showing that HMGB1 is involved in inflammation and oxidative stress. Moreover, HMGB1 and ROS are associated with NF-kB pathway, when siHMGB1 NAC were introduced, p-IKBα and p-p65 protein expression were effectively decreased, thus inhibiting the NF-kB-dependent gens transcription. Since NF-kB as mediator effect on inflammatory response [29, 38], above results further demonstrated that HMGB1 mediates LPS-induced inflammation in colon cancer cells.

On the other hand, besides being as a antioxidant enzyme, the current studies have shown that the activation of GPX4 helps to promote the inflammation resolution by eliminating the reactive oxygen species [39, 40]. Current studies have shown both HMGB1 and GPX4 contribute to inflammation, then we investigated the linkage of HMGB1 and GPX4, and the results showed that HMGB1 could interact with GPX4 and negatively regulated the GPX4 activity, while lacking of LPS-stimulated made HMGB1 fail to interact with GPX4. Under the LPS stimulated conditions, HMGB1 can export from nucleus to cytoplasm and Glycyrrhizic acid, the inhibitor of HMGB1, can block its translocation. Meanwhile, the levels of acetylated HMGB1 was significantly elevated, verifying that acetylated HMGB1 is responsible for interaction with GPX4. Thus our discoveries provided a novel mechanism for inflammation mediated by HMGB1.

Subsequently, by utilizing 50 pairs of colon tumor tissues, we analyzed the expression and correlation about HMGB1, GPX4 and p-p65, and then evaluated their correlation in colon cancer. The present study showed HMGB1 expression were positively correlated with GPX4 and p-p65, these clinical findings suggest the therapeutic targets for colon cancer.

## Conclusions

In conclusion, our results provided the evidences showing that acetylated HMGB1 can interact with GPX4, leading to oxidative stress and inflammation via NF-kB in colon cancer cells (Fig. 7). Further research is needed to understand how to reverse this effect to attenuate the ROS accumulation and inflammation. Taken together, our findings reveal a novel mechanism of HMGB1 in inflammation, providing therapeutic strategies for colon cancer.

**Fig. 7:** Schematic model for HMGB1 mediates LPS-induced inflammation via interacting with GPX4 in colon cancer cells

## Data Availability

The data that support the findings of this study are available from the corresponding author upon reasonable request.
